The article "Gemcitabine and cisplatin-induced tumor lysis syndrome in a patient with gallbladder carcinoma: A case report" was published in 2013. Journal: Oncol Lett.

# Gemcitabine and cisplatin-induced tumor lysis syndrome in a patient with gallbladder carcinoma: A case report

**DOI:** 10.3892/ol.2013.1189

**Published:** 2013-02-12

**Authors:** DEITER J. DUFF, SHADI HADDADIN, CARL FRETER, CHRIS PAPAGEORGIOU

**Affiliations:** 1 Departments of Pathology and Anatomical Sciences, University of Missouri School of Medicine, Columbia;; 2 Hematology and Oncology, University of Missouri School of Medicine, Columbia;; 3 SSM Cancer Care, St. Louis, MO, USA

**Keywords:** tumor lysis syndrome, gallbladder carcinoma, solid tumors, gemcitabine, renal failure

## Abstract

We report a case of tumor lysis syndrome (TLS) in a patient with gallbladder carcinoma. TLS has not been reported in association with this type of tumor. TLS typically occurs in cases of highly proliferative hematological malignancies and small cell carcinoma. Two factors that may have contributed to TLS in this case include multifactorial mild acute renal failure shortly before the administration of chemotherapy and the aggressive morphology of the gallbladder carcinoma, which was a poorly differentiated sarcomatoid variant. This case raises concern for the development of TLS in certain types of patients with solid tumors.

## Introduction

In the present study, we report a case of tumor lysis syndrome (TLS) in a patient with gallbladder carcinoma treated with gemcitabine and cisplatin. TLS occurs most commonly in highly proliferative hematological malignancies such as acute lymphoblastic leukemia, acute myeloid leukemia and Burkitt’s lymphoma (1). It also occurs in certain solid tumors, notoriously small cell carcinoma, and rarely in other types of tumor (2). Although TLS has been reported in hepatocellular carcinoma (2,3), to the best of our knowledge, this is the first reported case of TLS associated with gallbladder carcinoma.

TLS occurs when malignant cells lyse and release their contents, usually within 12–72 h of cytotoxic therapy (2,4,5). Release of intracellular contents leads to hyperuricemia, hyperphosphatemia, hypocalcemia and hyperkalemia. Laboratory TLS parameters have been suggested by Cairo and Bishop and include uric acid ≥8 mg/dl, potassium ≥6 mg/l, phosphorus ≥2.1 mmol/l (children) or ≥1.45 mmol/l (adults), and calcium ≤1.75 mmol/l, or a 25% change from baseline in any of these parameters (6). TLS is potentially fatal, possibly leading to renal failure or fatal arrhythmias (1).

Prevention is considered to be the best management and consists of aggressive intravenous fluids, allopurinol and rasburicase prophylaxis in high-risk patients (1). Although urine alkalanization has previously been used as treatment, it is no longer recommended by some groups as a viable treatment option (1). Instead, prevention treatment using these agents is now recommended.

The article "Gemcitabine and cisplatin-induced tumor lysis syndrome in a patient with gallbladder carcinoma: A case report" was published in 2013. Journal: Oncol Lett.

It has been suggested that the incidence of TLS in solid tumors is low (5), but it may be underestimated. A literature review found 45 reported cases, with a mortality rate of approximately 1 in 3 (2). In the present study, we demonstrate that even in the case of certain solid tumors, attention should be given to the possibility of a patient developing TLS.

The case report was approved by the Institutional Review Board at the University of Missouri.

## Case report

A 50-year-old male presented with abdominal pain. Laboratory tests showed mild leukocytosis (11,500/mcl) and anemia (11.7 g/dl). The patient had an elevated alkaline phosphotase of 152 U/l with otherwise normal liver function.

A computed tomography scan of the abdomen (Fig. 1) revealed a heterogeneous mass of the gallbladder fossa measuring 5×5×6 cm. There was also lymphadenopathy of periportal, pericaval, periaortic and mesenteric lymph nodes.

The gallbladder tumor was resected, but a curative resection was impossible due to massive lymphadenopathy of aortic, vena cava, and celiac areas. Final pathology revealed a 7-cm poorly differentiated adenocarcinoma with sarcomatoid features (Fig. 2). The tumor was found to have areas of brisk atypical mitoses. Lymph nodes showed metastatic adenocarcinoma.

The patient was diagnosed with a stage IV poorly differentiated adenocarcinoma of the gallbladder, AJCC stage IVB (T3 N2 MX0). The recommendation was a chemotherapy regimen of gemcitabine and cisplatin. Chemotherapy did not commence immediately due to poor performance status.

Approximately 2 weeks after this visit, the patient presented with shortness of breath and an inability to eat or drink. Laboratory test results on that day included a white blood cell count of 19,900/mcl, laboratory evidence of dehydration, total bilirubin of 3.4 mg/dl, alkaline phosphatase of 1652 U/l, AST 109 U/l, and ALT 40 U/l, a picture consistent with cholestasis. Due to tense ascites, paracentesis was performed. However, the patient also had elevated cardiac enzymes with possible ST elevations and Q waves. A cardiac catheterization showed single-vessel coronary artery disease, and medical therapy was recommended.

When his cardiac status had stabilized, a lengthy discussion was held with the patient. The decision was made to proceed with chemotherapy. The patient was administered one dose each of gemicitabine and cisplatin. On the second day after chemotherapy, the patient was dyspneic with air hunger. Urine output decreased to 300 ml over 24 h, even with high doses of IV lasix.

A diagnosis of tumor lysis syndrome was evident (Fig. 3). Laboratory results showed hyperkalemia (6.0 mmol/l), hyperphosphatemia (9.6 mg/dl), elevated uric acid (15.4 mg/dl) and evidence of acute renal failure with a creatinine of 2.69 mg/dl (previously normal). Corrected calcium was normal at 9.7 mg/dl, although ionized calcium was slightly reduced to a low of 1.06 mmol/l. The patient was treated with dialysis. His calcium-phosphorus product was 93 on the first day of dialysis, likely contributing to acute renal failure via nephrocalcinosis. His clinical picture was complicated by urosepsis, bilateral deep vein thrombosis and a possible pulmonary embolism. The patient succumbed 6 days after beginning chemotherapy to the disease.

The article "Gemcitabine and cisplatin-induced tumor lysis syndrome in a patient with gallbladder carcinoma: A case report" was published in 2013. Journal: Oncol Lett.

## Discussion

This is the first reported case of TLS developing in a patient with gallbladder carcinoma. There are at least two clinical factors that make this case unique and, in retrospect, increased the patient’s risk of TLS.

First, the patient had multi-factorial mild acute renal failure. He had mild contrast-induced nephropathy following cardiac catheterization, with creatinine increasing from a baseline of approximately 0.9 to 1.24 mg/dl the day after catheterization. It was also thought that volume depletion associated with paracentesis performed two days prior to the cardiac catheterization contributed to acute renal failure. These factors may have altered the patient’s renal function just enough to create a physiological condition favorable to the development of TLS. Pretreatment renal impairment is a reported risk factor for TLS in solid tumors, along with increased LDH and hyperuricemia (1,2).

Second, the tumor in this case was described as a poorly differentiated sarcomatoid type of adenocarcinoma. Brisk atypical mitoses were noted, indicating a highly proliferative tumor. This type of solid tumor may increase the risk of TLS compared to one that is slow-growing (fewer mitoses) and well-differentiated.

This raises the question of whether TLS prophylaxis such as allopurinol or rasburicase, urine alkalinization and intense hydration should be considered in certain types of solid tumors and/or in clinical situations such as in patients with mild acute nephropathy. Known risk factors for TLS include highly proliferative tumors (1,5), treatment-sensitive tumors, heavy tumor burden, and dehydration and/or renal disease (3). A recent expert TLS panel determined that the majority of solid tumors are in the low-risk category (4), but each clinical situation should be considered separately. TLS risk is particularly affected by renal function, and patients with low-risk tumors are moved into an intermediate risk category when renal dysfunction is present (4). It has been suggested that improvements in the treatment of some solid tumors, which were previously considered relatively insensitive to chemotherapy, have now rendered them more sensitive, thus placing these patients at a greater risk for TLS. As the mortality rate of patients with TLS in solid tumors may be higher than in patients with hematological malignancies (5), this renders prevention of TLS in certain solid tumors a clinical necessity (2,3).

The article "Gemcitabine and cisplatin-induced tumor lysis syndrome in a patient with gallbladder carcinoma: A case report" was published in 2013. Journal: Oncol Lett.

## Figures and Tables

**Figure 1:** Abdominal CT scan showed a heterogeneous gallbladder fossa mass invading the right hepatic lobe and enlarged periportal, pericaval, and periaortic lymph nodes.

**Figure 2:** Photomicrograph of tumor showing poorly differentiated adenocarcinoma with brisk mitoses and atypical tripolar mitosis (hematoxylin and eosin, magnification, ×200).

**Figure 3:** Graph of tumor lysis syndrome laboratory parameters.
